The article "Predefined Time Synchronization Control for Uncertain Chaotic Systems" was published in 2022. Journal: Comput Intell Neurosci.

# Predefined Time Synchronization Control for Uncertain Chaotic Systems

**DOI:** 10.1155/2022/3264936

**Published:** 2022-03-03

**Authors:** Yun Liu, Fang Zhu

**Affiliations:** ^1^School of Finance and Mathematics, Huainan Normal University, Huainan 232038, China; ^2^College of Science, Nanjing University of Aeronautics and Astronautics, Nanjing 211106, China

## Abstract

In this study, the predefined time synchronization problem of a class of uncertain chaotic systems with unknown control gain function is considered. Based on the fuzzy logic system and varying-time terminal sliding mode control technology, the predefined time synchronization between the master system and the slave system can be realized by the proposed control method in this study. The simulation results confirm the theoretical analysis.

## 1. Introduction

In recent decades, chaotic synchronization has been a research hotspot. The main reason is its wide application, such as in the fields of secure communication, biological systems, and so on [1–6]. Up to now, there are many synchronization methods between two chaotic systems, such as adaptive control [7–11], active control [12–14], impulsive control [15–17], and sliding mode control [18–23]. Among them, sliding mode control is deeply concerned by scholars because of its simple control principle and good robustness. Under the influence of unknown parameters and disturbances, two kinds of sliding mode synchronization methods were studied in [19]. Subsequently, to realize the state transient performance of the controlled system, many terminal sliding mode control methods were proposed. For example, a terminal sliding mode control method was employed in [22] and the synchronization of coronary artery system was realized. For fractional-order chaotic systems, [23] proposed a fractional-order terminal sliding mode control method, which synchronized two uncertain fractional-order systems. It should be pointed out that the initial value of the system should not be too far from the sliding mode; otherwise, the control performance will be affected. It should also be considered that the gain of the discontinuous controller should not be large, which will increase the serious chattering problem. In order to solve the above problems, a varying-time terminal sliding mode control method will be used to realize the predefined time synchronization of two uncertain chaotic systems.

In this study, the predefined time synchronization of the main system and the slave system is considered. The main highlights are as follows: the synchronization of two uncertain chaotic systems is realized by the varying-time sliding mode control method, and the case where the controller gain is unknown is considered. The rest of this study is organized as follows. Some preliminaries are given in Section 2. A preset time terminal sliding mode is proposed and main results are investigated in Section 3. A synchronization example is shown in Section 4. Finally, Section 5 gives a brief conclusion.

The article "Predefined Time Synchronization Control for Uncertain Chaotic Systems" was published in 2022. Journal: Comput Intell Neurosci.

## 2. Preliminaries

The master system is described as

(1) $$\begin{array}{c} \left\{\begin{array}{c} {\dot{\xi }}_{1}=\xi_{2},\\ {\dot{\xi }}_{2}=f_{1}\left(t,\xi_{1},\xi_{2}\right), \end{array}\right. \end{array}$$

where *ξ*_1_, *ξ*_2_ ∈ *ℝ* are the states of system (1), and *f*_1_(*t*, *ξ*_1_, *ξ*_2_) ∈ *ℝ* is a nonlinear function.

The slave system is described as

(2) $$\begin{array}{c} \left\{\begin{array}{c} {\dot{\eta }}_{1}=\eta_{2},\\ {\dot{\eta }}_{2}=f_{2}\left(t,\eta_{1},\eta_{2}\right)+g\left(t,\eta_{1},\eta_{2}\right)u, \end{array}\right. \end{array}$$

where *η*_1_, *η*_2_ ∈ *ℝ* are the states of system (2), *f*_2_(*t*, *η*_1_, *η*_2_) ∈ *ℝ* is a nonlinear function, *u* ∈ *ℝ* is the control input, and *g*(*t*, *η*_1_, *η*_2_) is a control gain function.

Define synchronization errors *e*_1_=*η*_1_ − *ξ*_1_, *e*_2_=*η*_2_ − *ξ*_2_. The aim of this study is to design a varying-time terminal sliding mode control method, so that the synchronization error *e*_1_ reaches a small neighborhood of zero in the predefined time. According to (1) and (2), one gets the synchronization error system as

(3) $$\begin{array}{c} \left\{\begin{array}{c} {\dot{e}}_{1}=e_{2},\\ {\dot{e}}_{2}=f_{2}\left(t,\eta_{1},\eta_{2}\right)-f_{1}\left(t,\xi_{1},\xi_{2}\right)+g\left(t,\eta_{1},\eta_{2}\right)u. \end{array}\right. \end{array}$$

In order to design the controller in this study, the following assumptions need to be made.

**Assumption 1 .**

States *ξ*_1_, *ξ*_2_, *η*_1_, *η*_2_ are measurable, and initial values *ξ*_2_(0)=*η*_2_(0).

**Assumption 2 .**

*f*_1_(*t*, *ξ*_1_, *ξ*_2_) and *f*_2_(*t*, *η*_1_, *η*_2_) are unknown but bounded.

**Assumption 3 .**

*g*(*t*, *η*_1_, *η*_2_) is unknown strictly positive and there exists a positive constant *χ*, such that *g*(*t*, *η*_1_, *η*_2_) > *χ*.

**Remark 1 .**

*ξ*_2_(0)=*η*_2_(0) in Assumption 1 is to ensure that the initial value of error system (3) belongs to the sliding mode, which will be designed later.  Assumption 2 ensures that the fuzzy logic system can be used to estimate the unknown function.

In order to achieve the aim of this study, the time-varying terminal sliding mode is considered:

(4) $$\begin{array}{c} z=\left\{\begin{array}{c} e_{2}+\beta e_{1}+2\lambda_{1}t+\lambda_{2}+\lambda_{3}{\left(e_{1}+\lambda_{1}t^{2}+\lambda_{2}t+\alpha \right)}^{q/p},\;t\leq T,\\ e_{2}+\beta e_{1}+\lambda_{3}e_{1}^{q/p},\;t>T, \end{array}\right. \end{array}$$

where *T* is a preset time, 0 < *q*/*p* < 1, *q* and *p* are the odds, *α*, *β* are the design positive constant, and *λ*_1_, *λ*_2_, and *λ*_3_ satisfy the following conditions:

(1) In order to ensure that the initial value of system (3) belongs to the sliding mode (4), i.e.,
  (5) $$\begin{array}{c} \beta e_{1}\left(0\right)+\lambda_{2}+\lambda_{3}{\left(e_{1}\left(0\right)+\alpha \right)}^{q/p}=0. \end{array}$$
(2) The sliding mode (4) is continuous at *t*=*T*, i.e.,
  (6) $$\begin{array}{c} \left\{\begin{array}{c} 2\lambda_{1}T+\lambda_{2}=0,\\ \lambda_{1}T^{2}+\lambda_{2}T+\alpha =0. \end{array}\right. \end{array}$$
(3) In order to ensure that sliding mode (4) can quickly approach the origin, i.e.,
  (7) $$\begin{array}{c} \lambda_{3}>0. \end{array}$$

Let

(8) $$\begin{array}{c} \Delta =\left\{\begin{array}{c} e_{1}+\lambda_{1}t^{2}+\lambda_{2}t+\alpha ,\;t\leq T,\\ e_{1},\;t>T. \end{array}\right. \end{array}$$

**Remark 2 .**

The article "Predefined Time Synchronization Control for Uncertain Chaotic Systems" was published in 2022. Journal: Comput Intell Neurosci.

The derivation of Δ^*q*/*p*^ with respect to time *t* may appear singular problem, and we modify $\Delta^{q/p-1}\dot{\Delta }$ as

(9) $$\begin{array}{c} \Delta^{q/p-1}\dot{\Delta }=\left\{\begin{array}{cc} \Delta^{q/p-1}\left(e_{2}+2\lambda_{1}t+\lambda_{2}\right) & ,\text{for }t\leq T\text{ and }\Delta \neq 0,\\ 0 & ,\text{for }t\leq T\text{ and }\Delta =0,\\ \Delta^{q/p-1}e_{2} & ,\text{for }t>T\text{ and }\Delta \neq 0,\\ 0 & ,\text{for }t>T\text{ and }\Delta =0. \end{array}\right. \end{array}$$

## 3. Main Result

Since *ξ*_1_, *ξ*_2_, *η*_1_, *η*_2_ are measurable, unknown functions *f*_1_(*t*, *ξ*_1_, *ξ*_2_), *f*_2_(*t*, *η*_1_, *η*_2_), and *g*(*t*, *η*_1_, *η*_2_) can be estimated by fuzzy logic systems [24, 25]. For *f*_1_(*t*, *ξ*_1_, *ξ*_2_), *f*_2_(*t*, *η*_1_, *η*_2_), and *g*(*t*, *η*_1_, *η*_2_), there exist *θ*_*f*_1__^*∗T*^*φ*_*f*_1__(*ξ*_1_, *ξ*_2_), *θ*_*f*_2__^*∗T*^*φ*_*f*_2__(*η*_1_, *η*_2_), and *θ*_*g*_^*∗T*^*φ*_*g*_(*η*_1_, *η*_2_), such that

(10) $$\begin{array}{c} \left\{\begin{array}{c} f_{1}\left(t,\xi_{1},\xi_{2}\right)=\theta_{f_{1}}^{*T}\varphi_{f_{1}}\left(\xi_{1},\xi_{2}\right)+\varepsilon_{f_{1}}\left(\xi_{1},\xi_{2}\right),\\ f_{2}\left(t,\eta_{1},\eta_{2}\right)=\theta_{f_{2}}^{*T}\varphi_{f_{2}}\left(\eta_{1},\eta_{2}\right)+\varepsilon_{f_{2}}\left(\eta_{1},\eta_{2}\right),\\ g\left(t,\eta_{1},\eta_{2}\right)=\theta_{g}^{*T}\varphi_{g}\left(\eta_{1},\eta_{2}\right)+\varepsilon_{g}\left(\eta_{1},\eta_{2}\right), \end{array}\right. \end{array}$$

where *ε*_*f*_1__(*ξ*_1_, *ξ*_2_), *ε*_*f*_2__*ε*_*g*_(*η*_1_, *η*_2_), and *ε*_*g*_(*η*_1_, *η*_2_) are the bounded fuzzy estimation errors, *θ*_*f*_1__^*∗T*^, *θ*_*f*_2__^*∗T*^, and *θ*_*g*_^*∗T*^ are the ideal weight vectors, and *φ*_*f*_1__(*ξ*_1_, *ξ*_2_), *φ*_*f*_2__(*η*_1_, *η*_2_), and *φ*_*g*_(*η*_1_, *η*_2_) are the Gaussian functions.

The article "Predefined Time Synchronization Control for Uncertain Chaotic Systems" was published in 2022. Journal: Comput Intell Neurosci.

From (3) and (4), the derivative of *z* with respect to *t* can be obtained as

(11) $$\begin{array}{c} \dot{z}=f_{2}\left(t,\eta_{1},\eta_{2}\right)-f_{1}\left(t,\xi_{1},\xi_{2}\right)+\beta e_{2}+g\left(t,\eta_{1},\eta_{2}\right)u\\ +\left\{\begin{array}{c} 2\lambda_{1}+\lambda_{3}\frac{q}{p}\Delta^{p/q-1}\dot{\Delta },\;t\leq T\\ \lambda_{3}\frac{q}{p}\Delta^{p/q-1}\dot{\Delta },\;t>T\; \end{array}\right.\\ =\theta_{f_{2}}^{*T}\varphi_{f_{2}}\left(\eta_{1},\eta_{2}\right)-\theta_{f_{1}}^{*T}\varphi_{f_{1}}\left(\xi_{1},\xi_{2}\right)+\beta e_{2}+\varepsilon_{f_{2}}\left(\eta_{1},\eta_{2}\right)\\ -\varepsilon_{f_{1}}\left(\xi_{1},\xi_{2}\right)+\theta_{g}^{*T}\varphi_{g}\left(\eta_{1},\eta_{2}\right)u_{e}+g\left(t,\eta_{1},\eta_{2}\right)u\\ +\left\{\begin{array}{c} 2\lambda_{1}+\lambda_{3}\frac{q}{p}\Delta^{p/q-1}\dot{\Delta },\;t\leq T,\\ \lambda_{3}\frac{q}{p}\Delta^{p/q-1}\dot{\Delta },\;t>T. \end{array}\right. \end{array}$$

Now, design the controller as

(12) $$\begin{array}{c} u=u_{e}+u_{s},\\ u_{e}=\frac{{\hat{\theta }}_{g}^{T}\varphi_{g}\left(\eta_{1},\eta_{2}\right)}{{\left({\hat{\theta }}_{g}^{T}\varphi_{g}\left(\eta_{1},\eta_{2}\right)\right)}^{2}+1}\left[\begin{array}{c} -{\hat{\theta }}_{f_{2}}^{T}\varphi_{f_{2}}\left(\eta_{1},\eta_{2}\right)+{\hat{\theta }}_{f_{1}}^{T}\varphi_{f_{1}}\left(\xi_{1},\xi_{2}\right)-k_{1}z-\beta e_{2}\\ +\left\{\begin{array}{c} -2\lambda_{1}-\lambda_{3}\frac{q}{p}\Delta^{p/q-1}\dot{\Delta },\;t\leq T\\ -\lambda_{3}\frac{q}{p}\Delta^{p/q-1}\dot{\Delta },\;t>T \end{array}\right. \end{array}\right]\\ ≜\frac{{\hat{\theta }}_{g}^{T}\varphi_{g}\left(\eta_{1},\eta_{2}\right)\Pi }{{\left({\hat{\theta }}_{g}^{T}\varphi_{g}\left(\eta_{1},\eta_{2}\right)\right)}^{2}+1},\\ u_{s}=-\frac{|\Pi |\text{sign}\left(z\right)}{\left({\left({\hat{\theta }}_{g}^{T}\varphi_{g}\left(\eta_{1},\eta_{2}\right)\right)}^{2}+1\right)\chi }, \end{array}$$

where *k*_1_ is a design positive constant, and ${\hat{\theta }}_{f_{1}}$, ${\hat{\theta }}_{f_{2}}$, and ${\hat{\theta }}_{g}$ are the estimations of *θ*_*f*_1__^*∗*^, *θ*_*f*_2__^*∗*^, and *θ*_*g*_^*∗*^. The parameter adaptation laws of ${\hat{\theta }}_{f_{1}}$ and ${\hat{\theta }}_{f_{2}}$ are given by

(13) $$\begin{array}{c} {\dot{\hat{\theta }}}_{f_{1}}=\gamma_{f_{1}}\left(-z\varphi_{f_{1}}\left(\xi_{1},\xi_{2}\right)-\delta_{f_{1}}{\hat{\theta }}_{f_{1}}\right),\\ {\dot{\hat{\theta }}}_{f_{2}}=\gamma_{f_{2}}\left(z\varphi_{f_{2}}\left(\eta_{1},\eta_{2}\right)-\delta_{f_{2}}{\hat{\theta }}_{f_{2}}\right),\\ {\dot{\hat{\theta }}}_{g}=\gamma_{g}\left(zu_{e}\varphi_{g}\left(\eta_{1},\eta_{2}\right)-\delta_{g}{\hat{\theta }}_{g}\right), \end{array}$$

where *γ*_*f*_1__, *γ*_*f*_2__, *γ*_*g*_, *δ*_*f*_1__, *δ*_*f*_2__, and *δ*_*g*_ are the design positive constants. Let *ε*(*t*)=*ε*_*f*_1__(*ξ*_1_, *ξ*_2_)+*ε*_*f*_2__(*η*_1_, *η*_2_)+*ε*_*g*_(*η*_1_, *η*_2_)*u*_*e*_. Obviously, *ε*(*t*) is bounded, i.e., there exists a positive constant *ε*^*∗*^, such that |*ε*(*t*)| ≤ *ε*^*∗*^.

The article "Predefined Time Synchronization Control for Uncertain Chaotic Systems" was published in 2022. Journal: Comput Intell Neurosci.

**Theorem 1 .**

Under Assumptions 1–3, if the time-varying terminal sliding mode (4), controller (12), and parameter adaptive laws (13) are employed, then all signals in (14) are bounded.

**Proof**

Consider the following Lyapunov function:

(14) $$\begin{array}{c} V_{1}=\frac{1}{2}z^{2}+\frac{1}{\gamma_{f_{1}}}{\tilde{\theta }}_{f_{1}}^{T}{\tilde{\theta }}_{f_{1}}+\frac{1}{\gamma_{f_{2}}}{\tilde{\theta }}_{f_{2}}^{T}{\tilde{\theta }}_{f_{2}}+\frac{1}{\gamma_{g}}{\tilde{\theta }}_{g}^{T}{\tilde{\theta }}_{g}, \end{array}$$

where ${\tilde{\theta }}_{f_{1}}=\theta_{f_{1}}^{*}-{\hat{\theta }}_{f_{1}}$, ${\tilde{\theta }}_{f_{2}}=\theta_{f_{2}}^{*}-{\hat{\theta }}_{f_{2}}$, and ${\tilde{\theta }}_{g}=\theta_{g}^{*}-{\hat{\theta }}_{g}$. From (11), derivation of *V*_1_ with respect to *t* yields

(15) $$\begin{array}{c} {\dot{V}}_{1}=z\dot{z}-\frac{1}{\gamma_{f_{1}}}{\tilde{\theta }}_{f_{1}}^{T}{\dot{\hat{\theta }}}_{f_{1}}-\frac{1}{\gamma_{f_{2}}}{\tilde{\theta }}^{T}{\dot{\hat{\theta }}}_{f_{2}}\\ =z\left[\begin{array}{c} \theta_{f_{2}}^{*T}\varphi_{f_{2}}\left(\eta_{1},\eta_{2}\right)-\theta_{f_{1}}^{*T}\varphi_{f_{1}}\left(\xi_{1},\xi_{2}\right)+\beta e_{2}+\varepsilon \left(t\right)\\ +\theta_{g}^{*T}\varphi_{g}\left(\eta_{1},\eta_{2}\right)u_{e}+g\left(t,\eta_{1},\eta_{2}\right)u_{s}\\ +\left\{\begin{array}{c} 2\lambda_{1}+\lambda_{3}\frac{q}{p}\Delta^{p/q-1}\dot{\Delta },\;t\leq T\\ \lambda_{3}\frac{q}{p}\Delta^{p/q-1}\dot{\Delta },\;t>T \end{array}\right. \end{array}\right]\\ -\frac{1}{\gamma_{f_{1}}}{\tilde{\theta }}_{f_{1}}^{T}{\dot{\hat{\theta }}}_{f_{1}}-\frac{1}{\gamma_{f_{2}}}{\tilde{\theta }}_{f_{2}}^{T}{\dot{\hat{\theta }}}_{f_{2}}-\frac{1}{\gamma_{g}}{\tilde{\theta }}_{g}^{T}{\dot{\hat{\theta }}}_{g}\\ =z\left[\begin{array}{c} {\tilde{\theta }}_{f_{2}}^{T}\varphi_{f_{2}}\left(\eta_{1},\eta_{2}\right)-{\tilde{\theta }}_{f_{1}}^{T}\varphi_{f_{1}}\left(\xi_{1},\xi_{2}\right)+\beta e_{2}+\varepsilon \left(t\right)\\ {\hat{\theta }}_{f_{2}}^{T}\varphi_{f_{2}}\left(\eta_{1},\eta_{2}\right)-{\hat{\theta }}_{f_{1}}^{T}\varphi_{f_{1}}\left(\xi_{1},\xi_{2}\right)+{\tilde{\theta }}_{g}^{T}\varphi_{g}\left(\eta_{1},\eta_{2}\right)u_{e}\\ +{\hat{\theta }}_{g}^{T}\varphi_{g}\left(\eta_{1},\eta_{2}\right)u_{e}+g\left(t,\eta_{1},\eta_{2}\right)u_{s}\\ +\left\{\begin{array}{c} 2\lambda_{1}+\lambda_{3}\frac{q}{p}\Delta^{p/q-1}\dot{\Delta },\;t\leq T\\ \lambda_{3}\frac{q}{p}\Delta^{p/q-1}\dot{\Delta },\;t>T \end{array}\right. \end{array}\right]\\ -\frac{1}{\gamma_{f_{1}}}{\tilde{\theta }}_{f_{1}}^{T}{\dot{\hat{\theta }}}_{f_{1}}-\frac{1}{\gamma_{f_{2}}}{\tilde{\theta }}_{f_{2}}^{T}{\dot{\hat{\theta }}}_{f_{2}}-\frac{1}{\gamma_{g}}{\tilde{\theta }}_{g}^{T}{\dot{\hat{\theta }}}_{g}. \end{array}$$

Substituting (12) and (13) to (15) yields

(16) $$\begin{array}{c} {\dot{V}}_{1}=-k_{2}z^{2}-\frac{z\Pi }{{\left({\hat{\theta }}_{g}^{T}\varphi_{g}\left(\eta_{1},\eta_{2}\right)\right)}^{2}+1}-\frac{g\left(t,\eta_{1},\eta_{2}\right)|z\||\pi |}{\left({\left({\hat{\theta }}_{g}^{T}\varphi_{g}\left(\eta_{1},\eta_{2}\right)\right)}^{2}+1\right)\chi }\\ +z\varepsilon \left(t\right)+\delta_{f_{1}}{\tilde{\theta }}_{f_{1}}^{T}{\hat{\theta }}_{f_{1}}+\delta_{f_{2}}{\tilde{\theta }}_{f_{2}}^{T}{\hat{\theta }}_{f_{2}}+\delta_{g}{\tilde{\theta }}_{g}^{T}{\hat{\theta }}_{g}\\ \leq -k_{2}z^{2}+z\varepsilon \left(t\right)+\delta_{f_{1}}{\tilde{\theta }}_{f_{1}}^{T}{\hat{\theta }}_{f_{1}}+\delta_{f_{2}}{\tilde{\theta }}_{f_{2}}^{T}{\hat{\theta }}_{f_{2}}+\delta_{g}{\tilde{\theta }}_{g}^{T}{\hat{\theta }}_{g}. \end{array}$$

Since the following inequalities hold:

(17) $$\begin{array}{c} z\varepsilon \left(t\right)\leq \frac{1}{4}z^{2}+\varepsilon^{*2},\\ \delta_{f_{1}}{\tilde{\theta }}_{f_{1}}^{T}{\hat{\theta }}_{f_{1}}\leq \frac{\delta_{f_{1}}}{2}\left(-{\tilde{\theta }}_{f_{1}}^{T}{\tilde{\theta }}_{f_{1}}+\theta_{f_{1}}^{*T}\theta_{f_{1}}^{*}\right),\\ \delta_{f_{2}}{\tilde{\theta }}_{f_{2}}^{T}{\hat{\theta }}_{f_{2}}\leq \frac{\delta_{f_{2}}}{2}\left(-{\tilde{\theta }}_{f_{2}}^{T}{\tilde{\theta }}_{f_{2}}+\theta_{f_{2}}^{*T}\theta_{f_{2}}^{*}\right), \end{array}$$

substituting (12) into ${\dot{V}}_{1}$ yields

(18) $$\begin{array}{c} {\dot{V}}_{1}\leq -\left(k_{1}-\frac{1}{4}\right)z^{2}-\frac{\delta_{f_{1}}}{2}{\tilde{\theta }}_{f_{1}}^{T}\theta_{f_{1}}-\frac{\delta_{f_{2}}}{2}{\tilde{\theta }}_{f_{2}}^{T}{\tilde{\theta }}_{f_{2}}+R^{*}, \end{array}$$

where *R*^*∗*^=*ε*^*∗*2^+*δ*_*f*_1__/2*θ*_*f*_1__^*∗T*^*θ*_*f*_1__^*∗*^+*δ*_*f*_1__/2*θ*_*f*_2__^*∗T*^*θ*_*f*_2__^*∗*^. Selecting *k*_1_, *δ*_1_, and *δ*_2_, such that *ı*_1_≜min{2*k*_1_ − 1/2, *γ*_*f*_1__*δ*_*f*_1__, *γ*_*f*_2__*δ*_*f*_2__} > 0, then

(19) $$\begin{array}{c} {\dot{V}}_{1}\leq -{ı}_{1}V_{1}+R^{*}. \end{array}$$

According to (19), we can conclude that all signals in (14) are bounded. This completes the proof.

The article "Predefined Time Synchronization Control for Uncertain Chaotic Systems" was published in 2022. Journal: Comput Intell Neurosci.

**Remark 3 .**

For *t* > *T*, $e_{2}={\dot{e}}_{1}=z-\beta e_{1}-\lambda_{3}e_{1}^{q/p}$, with the boundedness of *z*; there exists unknown constant *b*^*∗*^, such that |*z*| ≤ *b*^*∗*^. Let *V*_2_=1/2*e*_1_^2^, and one has

(20) $$\begin{array}{c} {\dot{V}}_{2}=e_{1}{\dot{e}}_{1}\\ =e_{1}\left(z-\beta e_{1}-\lambda_{3}e_{1}^{q/p}\right)\\ \leq -\left(\beta -\frac{1}{4}\right)e_{1}^{2}-\lambda_{3}e_{1}^{q/p-1}+b^{*2}. \end{array}$$

Let *β* > 1/4 and define

(21) $$\begin{array}{c} \Omega_{e}=\left\{e_{1}|\lambda_{3}e_{1}^{q/p-1}\leq \frac{b^{*2}}{1-\nu }\right\}, \end{array}$$

where *ν* ∈ (0,1). Obviously, if $e_{1}\bar{\in }\Omega_{e}$, ${\dot{V}}_{2}\leq -\lambda_{3}e_{1}^{q/p+1}+b^{*2}<-\lambda_{3}\nu e_{1}^{q/p+1}<0$, *V*_2_ will monotonically decrease only to enter Ω_*e*_. Therefore, we obtain the convergence range of the tracking error *e*_1_.

## 4. Numerical Simulations

In this section, the chaotic gyroscope system [26] is taken as an example to show the effectiveness of the proposed method (12). For the master system (1), define *f*_1_(*t*, *ξ*_1_, *ξ*_2_)=−10^2^(1 − cos  *ξ*_1_)^2^/sin^3^*ξ*_1_+sin  *ξ*_1_ − 0.5*ξ*_2_ − 0.05*ξ*_2_^3^+35.7  sin(2*t*)sin  *ξ*_1_. For the slave system (2), define *f*_2_(*t*, *η*_1_, *η*_2_)=−10^2^(1 − cos  *η*_1_)^2^/sin^3^*η*_1_+sin  *ξ*_1_ − 0.5*η*_2_ − 0.05*η*_2_^3^+35.5  sin(2*t*)sin  *η*_1_, *g*(*t*, *η*_1_, *η*_2_)=5+sin  *η*_2_. Obviously, *g*(*t*, *η*_1_, *η*_2_) > *χ*≜3. The initial values *ξ*_1_(0)=−1, *ξ*_2_(0)=1, *η*_1_(0)=2, and *η*_2_(0)=1. The fuzzy membership functions are selected as

(22) $$\begin{array}{c} \varphi \left(\rho \right)=\exp\left[-\frac{1}{2}{\left(\frac{\rho +7.5-2.5j}{1.2}\right)}^{2}\right], \end{array}$$

where *ρ*=*ξ*_1_, *ξ*_2_, *η*_1_, *η*_2_; *j*=1,2,3,4,5. First, select a group of parameters as *T*=2, *k*_1_=3, *q*=3, *p*=5, *β*=3, *α*=−5, *λ*_1_=−5/4, *λ*_2_=5, *λ*_3_=14/2^3/5^, and the simulation results are shown in Figures 1–3. Figures 1 and 2 show that the state *ξ*_1_ of master system (1) and the state *η*_1_ of slave system (2) are synchronized after *T*=2*s*. In order to overcome the influence of unknown gain *g*(*t*, *η*_1_, *η*_2_), Figure 3 shows that the controller *u* fluctuates at *T*=2*s*, and then, the controller has a small chattering phenomenon.

Extend the predefined time to *T*=5*s*, and parameters modify as *λ*_1_=−1/5, *λ*_2_=2, *λ*_3_=11/2^3/5^; other parameters remain unchanged. The simulation results are shown in Figures 4–6. Figures 4 and 5 show that states *ξ*_1_ and *η*_1_ are synchronized after *T*=5*s* (Figure 6). The controller *u* also has a small fluctuation at *t*=5*s*, and the chattering phenomenon is very small.

Obviously, the proposed control method (12) in this study can ensure the synchronization between master system (1) and slave system (2) at a predefined time and can also overcome the influence of unknown gain *g*(*t*, *η*_1_, *η*_2_).

The article "Predefined Time Synchronization Control for Uncertain Chaotic Systems" was published in 2022. Journal: Comput Intell Neurosci.

## 5. Conclusion

In this study, the predefined time synchronization problem of uncertain chaotic systems was investigated. The fuzzy logic system was used to estimate the unknown function. A time-varying sliding mode was constructed. The proposed varying-time terminal sliding mode control method in this study made all signals bounded and the synchronization error entered a small neighborhood of zero after the predefined time. Simulation results show the effectiveness of the method.

## Figures and Tables

**Figure 1:** Time response trajectory of *e*_1_ by using the proposed method (12) with *T*=2*s*.

**Figure 2:** Time response trajectories of *ξ*_1_ and *η*_1_ by using the proposed method (12) with *T*=2*s*.

**Figure 3:** Time response trajectory of controller *u* by using the proposed method (12) with *T*=2*s*.

**Figure 4:** Time response trajectory of *e*_1_ by using the proposed method (12) with *T*=5*s*.

**Figure 5:** Time response trajectories of *ξ*_1_ and *η*_1_ by using the proposed method (12) with *T*=5*s*.

**Figure 6:** Time response trajectory of controller *u* by using the proposed method (12) with *T*=5*s*.

## Data Availability

The datasets generated for this study are included within the article.
